The article "Effect and Mechanism of Flavored Tongxie Yaofang Decoction for Diarrheal Irritable Bowel Syndrome under Intestinal Microecology" was published in 2022. Journal: Evid Based Complement Alternat Med.

# Effect and Mechanism of Flavored Tongxie Yaofang Decoction for Diarrheal Irritable Bowel Syndrome under Intestinal Microecology

**DOI:** 10.1155/2022/3904571

**Published:** 2022-08-03

**Authors:** Shunyong He, Qiong Lin, Jianfeng Huang, Lin Zheng, Jinmei Lai, Chaoyuan Chen

**Affiliations:** The Affiliated People's Hospital of Fujian University of Traditional Chinese Medicine, Fuzhou 350004, Fujian, China

## Abstract

This research was to analyze the effect of flavored Tongxie Yaofang on diarrheal irritable bowel syndrome (IBS) by the situation of intestinal microecology. The treatment mechanism was analyzed, so as to provide a more effective treatment method for patients clinically. 60 IBS patients were selected as the research objects and were divided according to the different treatment methods. For the control group (*n* = 20 cases), oral pinaverium bromide tablets were given. For the treatment group (*n* = 40 cases), the flavored Tongxie Yaofang decoction was given in addition to conventional treatment. The curative effects on the two groups of patients were evaluated in combination with the changes in intestinal microecology. With the syndrome score, the total effective rate of the treatment group (92.5%) was obviously superior to the control group (80%) (*P* < 0.05). The clinical symptoms such as abdominal pain, abdominal distension, and diarrhea in the treatment group were significantly relieved after treatment in contrast to the control group (*P* < 0.05). Intestinal Bifidobacterium, *Escherichia coli*, and Bifidobacterium/*Escherichia coli* (B/*E*) ratio were all greatly higher than those in the control group (*P* < 0.05). In summary, flavored Tongxie Yaofang had a good effect in improving the symptoms of patients with diarrheal IBS and improved the microflora of Bifidobacterium and *Escherichia coli* in the intestinal tract of patients.

## 1. Introduction

Irritable bowel syndrome (IBS) is a functional disorder of the gastrointestinal tract, with the main clinical manifestations of gastrointestinal dysfunction accompanied by abdominal pain or discomfort, which are usually relieved after defecation [1]. According to clinical manifestations, it can be classified into diarrheal, constipated, mixed, and untyped IBS [2]. Diarrheal IBS refers to patients who had pasty/watery stools of more than 24% and lumpy/hard stools of less than 24%; it has a high incidence and a wide range of effects and is more common in young and middle-aged people [3]. It brings different degrees of negative impact on the work and life of patients [4]. The treatment of this disease in Western medicine relies on symptomatic treatment. But because the etiology and pathogenesis are not fully understood, patients are not satisfied with the current control of clinical curative effect and recurrence rate [5]. In contrast, traditional Chinese medicine (TCM) has particular advantages in improving symptoms [6]. Fan et al. (2017) [7] proposed that Tongxie Yaofang could significantly reduce symptoms, increase stool consistency, and reduce bowel movements in 4 weeks compared to Western medicine in the treatment of IBS [7]. Chen et al. (2018) [8] and Wang et al. (2020) [9] drew the same conclusion. However, the flavored Tongxie Yaofang refers to the addition and subtraction of drugs to the original prescription according to the clinical symptoms of patients. Its clinical effect is significant in the treatment of diarrheal IBS, and the curative effect is obviously better than that of Western medicine. However, there are fewer clinical research studies about flavored Tongxie Yaofang in the treatment of diarrheal IBS, and further study is needed.

The role of microecological changes in the pathogenesis of IBS has attracted the attention of experts in recent years. A study has revealed that the intestinal microbiome is important for normal gastrointestinal function and functions of other organs. Changes in the normal intestinal microbiome, dysbiosis, and changes in gut motility will lead to microbial overgrowth and altered gut permeability [10]. He et al. (2018) [11] propose that the gut is more susceptible to dysfunction and dysbiosis due to its contact with the external environment and gut microbes, which leads to intestinal inflammations, including IBS. It is of great significance of microecology in the pathogenesis of diarrheal IBS and to evaluate microecology to guide treatment. However, whether TCM can improve intestinal microecological changes in the treatment of diarrheal IBS needs to be explored.

This research was intended to provide more effective treatment methods for diarrheal IBS patients clinically. The curative effect of flavored Tongxie Yaofang decoction in diarrheal IBS was studied through intestinal microecological changes. Stool samples from patients were collected in both the control and treatment groups. The real-time fluorescent quantitative polymerase chain reaction (PCR) was adopted for detecting the intestinal Bifidobacterium and *Escherichia coli* in stool samples, as well as the logarithmic expression of paired and replicated deoxyribonucleic acid (DNA) in wet stools per g. Bifidobacterium and *Escherichia coli* in the intestinal tract were compared before and after treatment [12]. It was expected to improve the cure rate of diarrheal IBS patients clinically and reduce the recurrence rate.

## 2. Materials and Methods

### 2.1. Research Objects

Among patients admitted to The Affiliated People's Hospital of Fujian University of Traditional Chinese Medicine from February to December 2020, 60 patients with diarrheal IBS were included in this study. According to the different treatment methods, the patients were divided into a treatment group and a control group. The 20 patients in the control group were all treated with conventional Western medicine, and oral pinaverium bromide tablets were given. The 40 patients in the treatment group received the flavored Tongxie Yaofang decoction apart from conventional treatment through years of clinical experience. Combined with intestinal microecological changes, the curative effects of the two groups of patients were evaluated.

With the inclusion criteria, the included patients met the Western medicine diagnostic criteria of diarrheal IBS as well as the standards of TCM syndromes. They were 17–71 years old, having a course of disease of more than 1 year. They signed informed consent forms and were willing to receive the treatment. All the above criteria must be satisfied simultaneously. The exclusion criteria were formulated as follows. Patients did not meet the diagnostic criteria or the inclusion criteria. They took drugs that affect gastrointestinal motility, other antidiarrheal drugs, and antibiotics within 30 days before the treatment, or they were taking other drugs with stable efficacy. Pregnant women and lactating women were not included. Patients suffered from other organic diseases, tumors, or inflammatory bowel diseases of the digestive system, they had other organic diseases confirmed by colonoscopy or barium enema, or their diarrhea was caused by systemic diseases, such as lactase deficiency and hyperthyroidism. Patients had fever, anemia, and hematochezia, or they had severe metabolic disorders of heart, liver, kidney, or endocrine, hematopoietic disorders, malignant tumors, mental disorders, and other diseases in the acute phase. Patients disagreed to participate in this study, because they cannot tolerate the treatment for adverse reactions, or they cannot complete the treatment as required due to other reasons. Those that met any one of the above conditions were excluded. The following criteria were laid down for discontinuing clinical tests. Patients failed to stick with the treatment. Patients got serious adverse reactions or severe complications during the treatment. This study had been approved by the Medical Ethics Committee of The Affiliated People's Hospital of Fujian University of Traditional Chinese Medicine, and the family members of the patients included signed the consent forms.

### 2.2. Reagents and Instruments

Nucleic acid extraction reagents were purchased from Zhengzhou Zhijie Biotechnology Co., Ltd. Thermus aquaticus (Taq) enzymes were generated from a kit. Common chemical reagents were purely made in China.  Table 1 shows the main instruments used in this study.

### 2.3. Bacterial DNA Extraction from the Stools

The specimen was thawed and frozen at room temperature. 0.3 g stool was taken, and 1.1 mL phosphate buffer solution (0.06 mol/L, pH:7.5) was added to mix thoroughly for 6 minutes. The mixture was centrifuged at 1000 rpm for 1 min, and the supernatant was taken. The centrifugation and extraction were repeated 4 times. All the supernatants were collected and centrifuged at 14000 rpm for 1 min. The supernatant was removed, and the precipitation was retained. 1 mL phosphate buffer solution was added to mix the precipitation, and then it was centrifuged at 14000 rpm for 6 min. The supernatant was discarded, and the precipitation was washed 5 times with phosphate buffer solution. DNA purification was performed as follows. The bacterial fluid was centrifuged at 14000 rpm for 16 s, and a 200 *μ*L supernatant was taken as the isolate. 200 *μ*L DNA was extracted into a 0.6 mL centrifuge tube, and 51 *μ*L of the bacterial solution was added to the tube, reversed several times, and mixed well. It was placed for 4 min at room temperature. 25 pL DNA was added to extraction liquid B, reversed several times, and mixed thoroughly. It was centrifuged at 13000 rpm for 11 min, and the supernatant was still removed. 200 pL DNA was added to extraction liquid C, reversed repeatedly, and mixed well. It was centrifuged at 13000 rpm for 6 min, the supernatant was discarded, and the remains were put at room temperature or 56°C for 3–6 min to dry. 18 pL sample diluent was added to the suspension and centrifuged for a short time, and the liquid was dropped to the bottom of the tube. The supernatant was taken to generate the PCR.

### 2.4. Treatment Methods

The patients in the control group were given pinaverium bromide tablets (Abbott Laboratories Trading (Shanghai) Co., Ltd.) for symptomatic western medicine treatment, oral administration at 50 mg/time, 3 times/day. The patients in the treatment group were treated with years of clinical experience combined with flavored Tongxie Yaofang in addition to the symptomatic Western medicine treatment. The patients were conditioned by restricting the liver, strengthening the spleen, and correcting and activating blood circulation. The basic prescription of flavored Tongxie Yaofang was prescribed with the following medicine materials. It included 13 g Saposhnikovia divaricata, 16 g Atractylodes macrocephala koidz, 11 g dried tangerine peels, 16 g white paeony root, 16 g turmeric, 16 g Rhizoma corydalis, 1 g Costustoot, 1 g Lindera, and 31 g Jiubi. For patients with spleen deficiency, 16–31 g Codonopsis was added. For patients with abdominal murmur, 61 g dried ginger was added. For those with mucus in the stool, 1 g coptis was added. For those who had constipation with fewer defecations, 1 g betel nut was supplemented. For those with abdominal distension, 16 g dried green tangerine peels and 16 g Fructus aurantii were supplemented. For those who were often tired, 31 g Hairyvein agrimonia and 31 g root of Ficus hirta Vahl were supplemented. The decoction was given one dose per day for three consecutive weeks. The stool samples of all patients in the treatment group were taken before and after treatment, and their symptoms were recorded and scored before and after treatment. Patients in both groups were treated for 4 weeks.

### 2.5. Observation Indicators

The number of defecations per day of patients was recorded. It was in a severe grade if the patients had more than 6 defecations every day. It was moderate with 4-5 defecations, it was mild with 2-3 defecations, and it was normal with 1 defecation each day. For the stool characteristics, it was recorded as severe grade with mucus in stool and watery stool; it was moderate with mushy or a small amount of mucus. It was mild with soft or a small amount of mucus, and it was normal with striped stool. For abdominal pain, it was assessed as normal grade with no abdominal pain, and it was mild with mild or occasional pain. It was moderate with several times of pain a day, and it was severe with recurrent severe pain or colic. In terms of abdominal distension, it was assessed as normal, mild, moderate, and severe with no abdominal distension, occasional abdominal distension or that after eating, severe abdominal distension of up to 6.2 hours a day, and abdominal distension with bulge all the day, respectively.

With the scoring criteria, 0, 1, 2, and 3 points were recorded for normal, mild, moderate, and severe grades, respectively.

In clinical practice, a patient was cured as the symptoms and physical signs disappeared or basically disappeared, and the syndrome score decreased by greater than or equal to 95%. The curative effect was assessed as remarkably effective, as the symptoms and physical signs of the patient were obviously improved, and the syndrome score was reduced by greater than or equal to 70%. It was effective as the symptoms and physical signs were improved, and the syndrome score was reduced by greater than or equal to 30%. It was ineffective as the symptoms and physical signs were not improved or even worsened, and the syndrome score was reduced by less than 30%.

The calculation equation was expressed as follows: total effective rate = ((syndrome score before treatment − the score after treatment)/the score before treatment) x 100%.

### 2.6. Statistical Analysis

SPSS16 was used to complete statistics. The contents of intestinal Bifidobacterium and *Escherichia coli* were expressed by logarithmic values. The independent sample *T* test was adopted to compare the microecology before and after treatment in the treatment group and the control group. Paired *T*-test was used to compare the contents of Bifidobacterium and *Escherichia coli* and the syndrome scores of patients in the treatment group before and after treatment. The chi-square test was adopted for enumeration data.

## 3. Results

### 3.1. Comparison of General Data of the Patients

80 cases in total were selected for this study, and 20 patients who did not meet the requirements were excluded according to the exclusion criteria. Finally, 60 patients were included in this study and were divided into the treatment group and the control group with different treatment methods. As shown in Table 2, there was no significant difference in age and sex ratios of patients between the two groups (*P* > 0.05), showing the two groups were comparable in age and gender.

### 3.2. Improvement of Clinical Symptoms before and after Treatment

The evaluation results of abdominal pain, abdominal distension, and diarrhea in the patients in the two groups before and after treatment are shown in Tables 3–5. It was observed that the abdominal pain, abdominal distension, and diarrhea were significantly improved in patients in the treatment group, with statistically significant differences compared with those before treatment (*P* < 0.05). For patients in the control group, the abdominal pain and diarrhea were significantly improved compared with those before treatment, and the difference was statistically significant (*P* < 0.05) while the abdominal distension did not change significantly (*P* > 0.05) in patients in the control group. Compared with those in the control group, the clinical symptoms of patients in the treatment group were higher improved significantly, with statistically significant differences (*P* < 0.05).

### 3.3. Comparative Analysis of Clinical Curative Effects on Patients

Figure 1 shows the curative effect analysis of 40 patients in the treatment group. According to syndrome scores, it was cured, remarkably effective, effective, and ineffective in 10, 14, 13, and 3 cases. The total effective rate reached 92.5%. In the control group, it was cured in 2 cases, remarkably effective in 6 cases, effective in 8 cases, and ineffective in 4 cases, with a total effective rate of 80.0%. It suggested that flavored Tongxie Yaofang had a good clinical effect in treating diarrheal IBS.

### 3.4. Comparison of Intestinal Microecology before and after Treatment

The intestinal microbes of Bifidobacterium, *Escherichia coli*, and Bifidobacterium/*Escherichia* (B/E) of patients were compared before and after treatment between the two groups, and the results are shown in Figure 2. It was observed that there was no significant difference among Bifidobacterium, *Escherichia coli*, and B/E of patients between the control group and the treatment group before treatment (*P* > 0.05). Bifidobacterium, *Escherichia coli*, and B/E of patients in both groups increased significantly after treatment, suggesting the differences were statistically significant (*P* < 0.05). Compared with those in the control group, Bifidobacterium, *Escherichia coli*, and B/E of patients in the treatment group increased obviously, and the differences were also statistically significant (*P* < 0.05).

## 4. Discussion

Western medicine believes that diarrheal IBS is the result of a combination of multiple factors, which is related to abnormal gastrointestinal motion, visceral paresthesia, and psychological factors [13]. The clinical treatment of diarrheal IBS mainly depends on symptomatic treatment of western medicine, but the symptoms not the disease are cured, and the patients are prone to reoccurrence with a poor effect [14]. Clinical studies have discovered that the symptoms in most patients with diarrheal IBS cannot be relieved well [15]. Therefore, TCM treatment has attracted people's attention. TCM syndrome differentiation and treatment can not only improve symptoms but also shorten the course of diseases and relieve patients' suffering. It also has a notable effect on reducing the frequency of IBS [13]. Furthermore, some medical staff have found in the process of serving patients with diarrheal IBS that the Bifidobacterium and *Escherichia coli* in the intestinal tract of these patients are prominently increased [16]. The ratio of B/*E* can simply reflect the general situation of intestinal colonization resistance. However, diminished colonization resistance in the intestinal tract may also inhibit the growth and reproduction abilities of potential pathogens, such as Bifidobacterium, and maintain the function of the local immune system. This will result in local inflammations and erroneous release of chemical mediators and neurotransmitters [17, 18].

To learn the curative effect of flavored Tongxie Yaofang in the treatment of diarrheal IBS and the regulation of gastrointestinal microecological stability, this research was conducted. The total effective rate (92.5%) of the patients in the treatment group was greatly higher than that of the control group (80%) (*P* < 0.05). This suggested that the flavored Tongxie Yaofang through clinical syndrome differentiation could improve the curative effect in the symptomatic treatment. It had a good clinical effect on treating diarrheal IBS. Moreover, the relief of clinical symptoms such as abdominal pain, abdominal distension, and diarrhea in the treatment group was remarkably better in contrast to the control group (*P* < 0.05). This was consistent with the research results of Dai et al. (2018) [19]. The clinical curative effect of flavored Tongxie Yaofang was significantly greater than that of conventional drug therapy. In contrast, it could highly reduce abdominal pain scores, abdominal distension, diarrhea, defecation frequency, etc. This also indicated the great application prospect of TCM in treating diarrheal IBS. The research studies of Li et al. (2020) [20] and Yan et al. (2019) [21] also provided some support for this research, as immunohistochemistry was adopted to study the role of flavored Tongxie Yaofang in intestinal microecology in diarrheal IBS. The results showed that intestinal Bifidobacterium, *Escherichia coli*, and B/E ratios were observably higher in comparison with the control group (*P* < 0.05). It was revealed that the flavored Tongxie Yaofang could better improve gastrointestinal flora. However, the current related research studies are relatively lacking; thus, in-depth exploration is needed to verify the accuracy and representativeness of the results.

## 5. Conclusion

In this research, the curative effect of flavored Tongxie Yaofang in treating diarrheal IBS and the regulation of gastrointestinal microecological stability were explored. Thereout, it was concluded that the flavored Tongxie Yaofang had a better effect on relieving the symptoms of diarrheal IBS patients. It could also better regulate the microbial communities of Bifidobacterium and *Escherichia coli* in the patients' intestinal tract. However, the specific mechanism of Bifidobacterium and *Escherichia coli* in the pathogenesis of diarrheal IBS remained unclear. Therefore, it was necessary to prepare corresponding animal models for further exploration in the future. The sample size in this research was too small, and more experimental samples should be included. Clinical trials should be carried out in multicenter hospitals with larger samples, rather than in a single or small area. Anyhow, the application prospect of TCM in the clinical treatment of diseases was very impressive, and it was worthwhile for clinical workers to explore.

## Figures and Tables

**Figure 1:** Comparison of clinical curative effects between the two groups after treatment.

**Figure 2:** Changes in the intestinal microflora of patients before and after treatment. ^∗^ means *P* < 0.05 compared with those before treatment, while # means *P* < 0.05 compared with those in the treatment group.

**Table 1:** Major instruments used in this study.

Instruments	Production place
Table-top and high-speed refrigerated centrifuge	The United States

Fluorescent quantometer	Germany

Ultra-low temperature freezer	The United Kingdom

Biosafety cabinet	Japan

**Table 2:** General data of the patients.

Groups	Sample size	Average age (years)	Male (cases)	Female (cases)
Treatment group	40	42.13 ± 11.12	28	12
Control group	20	33.76 ± 6.34	14	6
Statistic value	—	0.443	−0.325	
*P*	—	0.268	0.488	

**Table 3:** The severity of abdominal pain before and after treatment.

	Treatment group (*n* = 40)				Control group (*n* = 20)			
	Normal	Mild	Moderate	Severe	Normal	Mild	Moderate	Severe
Before treatment	6	26	4	4	1	15	3	1
After treatment	22^*∗*^	18	0	0	3	15	2	0
Statistic value	4.557				1.135			
*P*	0.000				0.043			

Note: ^*∗*^ suggested *P* < 0.05.

**Table 4:** The severity of abdominal distension before and after treatment.

	Treatment group (*n* = 40)				Control group (*n* = 20)			
	Normal	Mild	Moderate	Severe	Normal	Mild	Moderate	Severe
Before treatment	16	22	2	0	8	10	1	1
After treatment	30^*∗*^	10	0	0	8	12	0	0
Statistic value	3.289				0.097			
*P*	0.000				0.553			

Note: ^*∗*^ indicated *P* < 0.05.

**Table 5:** The severity of diarrhea before and after treatment.

	Treatment group (*n* = 40)				Control group (*n* = 20)			
	Normal	Mild	Moderate	Severe	Normal	Mild	Moderate	Severe
Before treatment	4	26	10	0 ^*μ*^	2	13	5	0
After treatment	32^*∗*^	6	2	0	5	12	2	1
Statistic value	5.569				1.436			
*P*	0.000				0.038			

Note: ^*∗*^ indicated *P* < 0.05.

## Data Availability

All data generated or analyzed during this study are included in this article.
